# Automatic Text Summarization for Public Health WeChat Official Accounts Platform Base on Improved TextRank

This article has been retracted.

**DOI:** 10.1155/2022/1166989

**Published:** 2022-07-13

**Authors:** Zixuan Cheng, Shunli Guo

**Affiliations:** ^1^School of Electronic and Information Engineering, Changchun University, Changchun 130022, China; ^2^School of Media, Qufu Normal University, Rizhao 276826, China

## Abstract

With the rapid development of we-media information dissemination, WeChat official accounts platform has become an important way for people to obtain health related knowledge. However, the platform information is redundant, miscellaneous, and overloaded. In order to meet the increasingly accurate and efficient knowledge service needs of users, reorganizing and aggregating document knowledge resources is effective. If we use the way of artificial recognition to filter information, it will inevitably cause huge labor and time cost, and the effect is very little in front of massive articles. This paper proposes a text summarization method for the WeChat platform based on improved TextRank that takes into account both user demands and sentence features during the summarization process. The data source crawled from the Sogou WeChat platform. The results show that the TextRank algorithm has obvious hints on the accuracy of text summarization extraction after fusing the Word2vec model. The improved TextRank method, integrating user demands and sentence features into the model, makes the results of text summarization closer to the theme of the article and more able to meet the user demand. According to the complexity of the algorithm, this method is not suitable for the automatic summarization of long or multiple documents.

## 1. Introduction

In the era of the mobile Internet, social media represented by microblogs, WeChat, and short-form videos has become a part of people's lives. However, social media addiction can lead to health problems such as burning eyes, headaches, and sleep disorders [1, 2]. WeChat official accounts platform remains China's most iconic mobile application and has quickly become the mainstream media for spreading health knowledge. The total number of articles published by public health WeChat official accounts such as “Dingxiang Doctor,” “Good Doctors,” “Family Doctors,” and “Hua Yi Wang” can reach more than 5 million times per week. The research shows that the user knowledge demands of the WeChat platform are high-quality integrated and rich in knowledge resources, multifunctional beautiful interface, and reliable system, as well as intelligent and personalized service [3]. However, most of the titles of the current articles on the platform are intended to attract attention, while a few titles indicate the theme of the text. There will be a misunderstanding to speculate the content by the title of the text. Therefore, how to identify effective information from a wide range of message push and improve reading efficiency has become an urgent need for WeChat users. The summary is a brief and accurate description of the important content of the literature. Without comments and supplementary explanations, it can summarize the core ideas of the text since the WeChat platform does not specify the format of the information, and many texts do not have introductions or summaries. The automatic summarization of knowledge resources on the WeChat platform can effectively solve the contradiction between knowledge redundancy and the limited reading ability of users and provide users with high quality and integrated information [4]^.^

At present, the research on health information of WeChat official accounts platform mainly focuses on the influence of the WeChat platform on the rehabilitation of certain diseases [5, 6], the sharing behavior of health information through WeChat [7], the promotion of WeChat platform on health information education [8, 9], and knowledge service improvement method based on label aggregation [4]. Few studies on improving the information service of the WeChat platform by automatic text summarization. This paper proposes a text summarization method for the WeChat platform based on improved TextRank, which comprehensively considers user demands and sentence features in the process of summarization. Introducing automatic summarization into the knowledge service of the WeChat platform can effectively concentrate knowledge content, improve user reading efficiency, improve knowledge reuse efficiency of the platform, and provide a better reading experience for health information users of WeChat official accounts.

## 2. Related Work

### 2.1. WeChat Official Account Platform

WeChat is an instant messaging service application launched by Tencent in 2011. It has become an indispensable part of people's communication, social, entertainment, and life. At present, the number of active users has reached 1.2 billion. Tencent launched its platform function on WeChat for the first time in July 2012, which made WeChat a public platform as a new form of media penetrating into emotion, people's livelihood, finance, culture, science and technology, and other fields. WeChat users can read, forward, praise, and comment on the platform's content. It has evolved into an important channel for people to exchange and disseminate information on a daily basis.

#### 2.1.1. Forms of Knowledge Resources on the WeChat Platform

The forms of the WeChat platform supporting push messages include text, voice, pictures, recordings, graphic messages, business cards, videos, and so on. A variety of content forms can coexist in a group of messages. There are few articles published by the WeChat public platform in the form of single media, which are generally text-based graphic messages. In some articles, background music or simultaneous reading pronunciation is inserted to make the content more abundant.

#### 2.1.2. Knowledge Types of Public Health WeChat Official Accounts

According to the different professional depths of knowledge, public health WeChat platform knowledge can be divided into popular science knowledge, professional popular science knowledge, professional frontier knowledge, professional knowledge, and academic topic knowledge. The audience of popular science knowledge is the most extensive, which plays a positive role in promoting knowledge popularization. The audience of professional popular science knowledge is also very wide. The attention of ordinary users to such knowledge varies according to the heat of the field, and the professional popular science knowledge in health and finance is paid more attention. The knowledge of professional frontiers, professional knowledge, and academic topics has certain requirements for the basic knowledge of WeChat users, so the audience is relatively small. The audience is mainly graduate students, university teachers, and scientific researchers.

#### 2.1.3. Characteristics of Knowledge Resources on the WeChat Platform

First of all, WeChat public account knowledge resources present fragmentation characteristics suitable for fragmentation reading. Due to the fast pace of life, fragmented reading has become the mainstream reading mode. Knowledge types and communication forms on WeChat official accounts are in line with the needs of modern people and the development trend of the times.

Secondly, higher requirements are also put forward for the quality of knowledge resources in refining, decomposing, restructuring professional knowledge content, and deducing it in a simple way. However, the current knowledge content of the platform is mainly generated by WeChat official accounts. There is a problem that the quality of knowledge is not high, and there are even many false, which brings trouble to users' reading.

In addition, there is a lot of information redundancy in the WeChat platform. There are a large number of WeChat official accounts, but some lack originality. Hot topic articles with similar content are frequently pushed by different official accounts. A frequent push of similar articles is a waste of information resources. At the same time, users' efficient fragmented reading time is constantly wasted on repetitive articles. Therefore, how identifying effective information from a wide range of message push and improve reading efficiency has become an urgent demand for WeChat users.

### 2.2. Automatic Text Summarization

Because of the massive amount of textual content that grows exponentially on the Internet and the various archives of news articles, scientific papers, legal documents, and so on. Automatic Text Summarization (ATS) is becoming increasingly important. Manual text summarization takes a lot of time, effort, and money, and it becomes impractical when dealing with massive amounts of textual content [10]. This paper studies the single text automatic summarization released by WeChat official accounts platform. Extractive and abstractive summarizations are the two types of automatic summarization. Extractive summarization extracts the article's original sentences with high weight without modifying the sentences and organizes the sentences in a certain order [11]. At the same time, abstractive summarization is to organize and generate new sentences after understanding the original text to describe the theme and main information [12]. Given the difficulties of language expression and information fusion, abstractive summarization is more complex and difficult than extractive summarization. More above, the extractive method selects sentences from the original text, which has low grammatical and syntactic error rate. Therefore, this paper adopts the extraction summarization to summarize the test of the WeChat platform.

How to judge the importance of sentences is a key problem to be solved in the extraction method [13]. In the beginning, sentence weight calculation was based on word frequency that the more frequent the words appear, the higher the weight of the words is. Sentences with more high-frequency words are more important. Sentence position, headline, cue words, and other features were gradually incorporated into the calculation of sentence weight in further research [14]. Salon proposed a method based on TFIDF, which effectively identified high-frequency invalid words by introducing an external background corpus and improved the effect of summarization [15]. However, language is a complex network [16], and the statistical-based methods cannot reflect complex relations such as syntax, grammar, and semantics. In view of this, an automatic summarization based on a graph model was proposed. It took words, sentences, and the relationships between them as nodes and edges to establish the corresponding network of graph model, then identified important sentences. The related algorithms include PageRank, LexRank, and TextRank [17–19]. The model, without any other statistical characteristics of sentences, achieved good results in the third place in the 15 comparison systems [19]. Due to the superiority of the graph model algorithm, it has been widely used in automatic summarization.

### 2.3. Automatic Text Summarization Base on TextRank

TextRank algorithm is a sort algorithm based on a graph model and a common method of text mining. The main idea of automatic summarization is sorting, that is, calculating and sorting the importance of sentences and extracting the sentences with the highest sorting as the content of the document summary. Similarly, the basic idea of automatic text summarization based on TextRank is to divide the text into sentences and establish a graph model. The voting mechanism is used to sort the sentences in the text according to their weight, and the top-ranking sentences are selected as a result. First, the text is preprocessed, and the word set of each sentence is composed of nodes of the graph model. The edge weight of the graph model is then used to calculate the degree of similarity between sentences. Construct a graph model and iteratively calculate sentence node weight. The iterative calculation formulas as shown in the following formula:

(1) $$\begin{array}{c} WS\left(V_{i}\right)=\left(1-d\right)+d\sum_{\left(j,i\right)\in \varepsilon }V_{j}\in In\left(V_{i}\right)\frac{w_{ji}}{\sum v_{k}\in Out\left(V_{j}\right)w_{jk}}WS\left(V_{j}\right), \end{array}$$

where *WS*(*V*_*i*_) represents the weight of the sentence *V*_*i*_, and *w*_*ij*_ represents the similarity between sentences *V*_*i*_ and *V*_j_, the summation represents the contribution of each adjacent sentence to the sentence. *In*(*V*_*i*_) represents a set of all sentence nodes pointing to node *V*_*i*_, *Out*(*V*_*i*_) represents a set of sentence node *V*_*j*_ pointing to sentence nodes, *d* represents a damping coefficient of 0.85. Finally, according to the sentence weight values to extract important N sentences as text summaries. The process of automatic text summarization based on TextRank is shown in Figure 1.

The traditional TextRank method's main flaw is that it only considered the correlation between sentences and did not integrate the important attribute of text sentence features. When constructing the edge weight value of the text graph model, the sentence similarity was calculated by calculating the frequency of cooccurrence words between sentences, which only considered the cooccurrence relationship between words and ignored the semantic relationship. Based on the existing research results, this paper improved the TextRank method by introducing external background corpus and sentence features. The Word2Vec model was integrated into the text vectorization expression, and the important sentence features such as user requirements, sentence location, and title similarity were considered in the algorithm. Automatic text summarization of public health WeChat official accounts used improved TextRank.

## 3. Automatic Text Summarization Based on Improved TextRank

In this paper, the traditional TextRank algorithm was optimized. Firstly, the Word2Vec model was used for text vectorization. Text title, content, and user demand were vectorized, respectively. The improved TextRank took sentences as nodes and the similarity matrix of nodes as the edge of the graph model. The initial weight and edges of the graph model were adjusted based on TextRank by calculating the similarity between sentences, the similarity between sentences and titles, the similarity between sentences and user demands, and the location information of sentences. Then iteratively compute the weight of nodes based on TextRank. The weights of nodes were sorted to form the final text summary. The process of single text summarization for the WeChat official accounts platform is shown in Figure 2.

### 3.1. Sentence Vectorization Based on Word2vec

The TextRank method takes the similarity between sentences as the edge to establish a graph model, which calculates the cooccurrence relationship between words in sentences. However, the study found that computing semantic similarity between sentences can get a better summary extraction effect [20]. Semantic similarity calculation has long been a challenge in natural language processing. Edit distance calculation, Jaccard coefficient calculation, chord similarity calculation, TFIDF calculation, and word vector average calculation are currently the most commonly used sentence similarity calculation methods. Semantic similarity between sentences refers to the semantic similarity of sentences. Sentences are composed of words or phrases according to a certain grammatical structure. Each sentence is a whole, and its similarity is based on the similarity of words. In order to calculate the semantic similarity of sentences, this paper introduces the Word2vec word vector model for text vectorization.

Mikolov proposed Word2vec [21] in 2013 as a model for training word vectors, and it has since been widely used in a variety of text mining tasks. It can effectively solve the high dimensional problem of traditional word vector representation by mapping each word to a relatively low dimensional vector space. The Word2vec model has two training modes: CBOW and Skip-Gram. The CBOW model principle is to predict the current word using context words, whereas the Skip-Gram model predicts context words using current words. WeChat platform knowledge resources are huge, and abstract extraction in most cases for high-frequency words in the text, so this paper selects the CBOW model for training.

The corpus is trained first, and then the word vector representation of the corpus is obtained. Averaging the word vector yields the sentence vector. To achieve better semantic similarity results, it uses the similarity between sentences as the edge weight of the graph. In addition, the use of a large number of external background corpus in the training of Word2vec model also helps to improve the effect of summarization.

### 3.2. Sentence Features Calculation

When extracting sentences to generate a summary, the TextRank algorithm only considers the similarity between the sentences in the graph nodes, disregarding all other factors. The algorithm is improved in this paper based on the writing habits of Chinese text, and the characteristics of the position and title similarity of the text where the sentence is located are fully considered. Specific sentence features influence and quantitative methods are as follows.

#### 3.2.1. Sentence Location and Quantization

Sentence position refers to the sentence's position in the text paragraph, which has a significant impact on the importance of the sentence, particularly the sentence at the end of the article [22]. The study has shown that the probability that the first sentence of the paragraph was selected as a summary exceeds 85% and that the sentence at the end of the paragraph was also selected as a summary accounts for nearly 70% [23]. The first sentence or the first paragraph in the articles on the WeChat platform is called the introduction, which requires a high degree of summary of the content. Therefore, this paper improved the initial weights of the first sentence and the last sentence in the text. When the sentence is at the beginning or end of the paragraph, the sentence weight correction formula is shown in the following formula:

(2) $$\begin{array}{c} WS\left(V_{i0}\right)=WS\left(V_{i0}+\text{e}\right), \end{array}$$

where *WS*(*V*_*i*_) is the initial weight of the sentence, *WS*(*V*_*i*0_) represents the weight adjusted by the position feature relationship, *e* ∈ (0,1) represents the correction coefficient.

#### 3.2.2. Similarity Calculation of Title and Sentence

For Chinese writing habits, the title is often highly summarized for the full text. The sentence with high similarity to the title has a greater possibility of becoming the final summary sentence. As a result, the similarity between sentences and the title in the text was calculated, and the initial weight of sentence nodes in the graph model was modified. The similarity between the text title and the sentence is calculated. If the similarity is high, the initial weight of the sentence would be modified. The rules of modification are shown in the following formula:

(3) $$\begin{array}{c} \left\{\begin{array}{cc} \text{WS}\left(V_{i0}\right)=\text{WS}\left(V_{i0}\right)+\text{sim}T, & 0.5<\text{sim}T\leq 1,\\ \text{WS}\left(V_{i0}\right)=\text{WS}\left(V_{i0}\right), & 0\leq \text{sim}T\leq 0.5, \end{array}\right. \end{array}$$

where *WS*(*V*_*i*0_) represents the weight adjusted by the sentence location, sim*T* represents the value of semantic similarity between the title and the sentence, the threshold of which is set to 0.5.

#### 3.2.3. The Similarity Calculation of User Demand and Sentence

The knowledge service of the WeChat platform is user-oriented, and the ultimate goal is to meet the needs of users. Different user groups may have different information contents and concerns for the same document. Based on TextRank automatic summarization, the sentences are extracted to form a summary ‘one thousand people one face' without considering the user's characteristics and personalized knowledge needs. In order to meet the needs of users, this paper made text vectorization of the user request and extracted sentences with high similarity to user requests as summary sentences. It is considered that sentences with high similarity to users' needs can better express what users want to know. Therefore, this paper calculates the similarity between each sentence in the text and the user requests and then modifies the initial weight of the sentence node in the graph model. The calculation and modification rules of user requests are similar to the title shown in (2).

## 4. Experimental Results and Analysis

### 4.1. Data Acquisition and Pretreatment

The experimental data in this paper are derived from the big data platform of Qingbo Index, which provides big data mining, big data analysis, and public opinion analysis services. We selected the top 10 accounts articles in the WeChat official accounts “China Health” list, including “DingXiangYiSheng,” “DingXiangLab,” “bjcdcblog,” “huayiwang91,” “mengzhuariji,” “jtys1983,” “WestChina_Hospital,” “srrsh199405,” “vom120,” and “Health Care.” The top 10 articles, within one month from May 5 to June 5 in 2022, in each WeChat official account reading list were collected, a total of 100 articles. Each document included the title and text of the articles. Removed documents that were too long, too short, or less knowledgeable, and finally selected 50 to form the experimental corpus.

Because the articles on the WeChat platform are network documents, there are redundant and different media formats, and the summary generally includes only text. Firstly, pretreatment of the experimental corpus by removing nontext class labels such as special characters, formulas, pictures, tables, hyperlinks, etc. Then, using python's Jieba package for word segmentation and sentence segmentation, the shortest text had 12 sentences, the longest text had 78 sentences, and the average length was 46 sentences. The content of the sentence number 0 was set as user requests, the content of sentence number 1 was the title of the document, and the sentence after number 2 was the rest of text. At last, extracted sentences by 20% compression.

### 4.2. Performance Comparison

In order to verify the effectiveness of the automatic text summarization method for articles in public health WeChat official accounts proposed in this paper, the summary results extracted by the Improved TextRank, TextRank, Word2vec + TextRank, and MMR were compared and analyzed. Due to the small scale of an experimental corpus, the Edmundson method was used to evaluate the effect of text summarization that calculated the average coincidence rate P between automatic text summarization and manual summarization, as shown in the following formula:

(4) $$\begin{array}{c} P=\frac{\sum_{i=1}^{n}\left(\left|S_{i}\cap R_{i}\right|/\left|S_{i}\right|\right)}{n}, \end{array}$$

where *S*_*i*_ represents the summary sentence sets generated by automatic summarization of text *i*, *R*_*i*_ represents the summary sentence sets generated by manual summarization of text *i*, and *n* represents the total number of texts.

Taking the articles ‘After 17 times of nucleic acid negative diagnosis, experts responded: the problem may be…' released by “huayiwang91” on June 2 as an example, assumed user requirements was that ‘the reasons for multiple nucleic acid negative but confirmed.' Out of a total of 33 sentences, 6 sentences were extracted as a summary. Four methods were used for summary extraction, and the results were compared with the manual results. The comparison results are shown in Table 1 The sentences in the shadow section are consistent with the results of the artificial summary.

Comparing the average value of *P* of four automatic summarization methods when extracting 4, 6, 8, and 10 sentences, respectively, with experimental corpus, the results were shown in Table 2.

### 4.3. Discussion and Analysis

According to the data in Table 1, the coincidence rate of the Improved TextRank method reached 4/6, which was much better than that of the method based on TextRank (1/6). Although, compared with the methods based on MMR and word2vec + TextRank, the advantage of coincidence rates of Improved TextRank was not obvious.

Through the data analysis in Table 2, the average coincidence rate in terms of *P* of the summary extracted by the automatic text summarization based on Improved TextRank in this paper increased as the number of extracted sentences increased. When the number of sentences reached 10, the accuracy decreased, indicating that the method is more suitable for short text summarization extraction. The automatic text summarization based on Improved TextRank and word2vec + TextRank, whose average coincidence rate *P* reached 60% or less, outperformed the other two methods. It demonstrates that incorporating the Word2vec word vector model significantly improved extraction accuracy. However, by comparing summaries of Improved TextRank and word2vec + TextRank, it is found that after fusing user demands and sentence features, the summaries can semantically better express the theme of the article. At the same time, considering the users' request in the method, summaries could better match users demands, which enable summary extraction to meet user-oriented personalized demands.

The experimental results showed that the automatic text summarization based on the Improved TextRank, considering the factors of user requirements, titles, and the sentence features during the extraction process, the readability, accuracy, and quality of the summary were improved.

## 5. Conclusion

WeChat official accounts platform provides public health information for more and more users. Users also put forward higher requirements for information services. Improving the information dissemination efficiency of the WeChat platform is of great significance to health knowledge dissemination. As an important form of knowledge integration organization, automatic summarization technology can help users quickly understand the content of the article in a short time. In the age of big data, it can effectively solve the problem of knowledge overload in WeChat official accounts and reorganize knowledge resources for the innovative knowledge service mode of the WeChat platform. This will meet the increasingly precise and intelligent service demands of users. Based on the TextRank, this paper attempted to train the Word2vec model by introducing external background corpus and deeply excavating the relationship between sentences. When initializing the graph model, multiple sentence features such as sentence position, title similarity, and user demand similarity were considered. The feasibility and effectiveness of the automatic summarization method proposed in this paper were validated through the collection of ten WeChat official accounts for experimental research. The experimental results showed that the introduction of the Word2vec model can improve the accuracy of summary extraction as a whole; considering sentence features can make the extracted summary better to meet user demands. Based on the summary of text on the WeChat platform, the knowledge integration service model is proposed to meet the service needs of users to obtain integrated and personalized knowledge efficiently and conveniently.

In the choice of sentence features, this paper focused on the factors such as sentence location, title similarity, and user needs. In fact, it can also integrate the factors such as sentence length and general tagging words to further optimize the algorithm. The automatic summarization method proposed in this paper is appropriate for WeChat platform text and text of similar length. Since the number of sentences is too large and the training word vector model is too complex, for automatic summarization of multidocuments, text vectorization of sentences and paragraphs can be considered, such as the Doc2Vec model.

## Figures and Tables

**Figure 1:** Automatic text summarization of WeChat based on TextRank.

**Figure 2:** Automatic text summarization of WeChat based on Improved TextRank.

**Table 1:** The example of automatic summarization.

Method and coincidence rate	Summary
Manual	Recently, Changping District of Beijing reported that a woman was diagnosed after 17 nucleic acids were negative in May, which attracted the attention of internet users. Throughout the two years of the epidemic, this kind of event was not an example. After multiple nucleic acids were negative, the diagnosis was still confirmed. Here are the experts responses.
	There have been multiple nucleic acid negative confirmed cases through information collection, and we it is not difficult to find that multiple nucleic acid negative confirmed cases are not rare.
	Second, after multiple nucleic acid negative diagnoses, expert response: normal phenomenon, can understand the face of more and more cunning variant strains.
	The virus may not be present at the site of the test.
	Third, virus mutation immune escape drive increases or increases the difficulty of nucleic acid screening.
	The weekly report pointed out that the related variation may affect the characteristics of BA. 5, making it appear to have a growth advantage over BA. 1 and BA. 2, which may be mainly driven by immune escape.

Improved TextRank (4/6)	Recently, the Changping District of Beijing reported that a woman was diagnosed after 17 nucleic acids were negative in May, which attracted the attention of internet users. Throughout the two years of the epidemic, this kind of event was not an example. After multiple nucleic acids were negative, the diagnosis was still confirmed. Here are the experts' responses.
	There have been multiple nucleic acid negative confirmed cases through information collection, and it is not difficult to find that multiple nucleic acid negative confirmed cases are not rare.
	Occasionally, at the beginning of this year, the office of the new coronal pneumonia epidemic prevention and control command of Zhengzhou city also disclosed a similar confirmed case, and the local no. 96 case was finally diagnosed after seven nucleic acid tests for seven consecutive days.
	At the same time, after relevant media investigation, before this, Xi'an has also shown seven nucleic acids after the diagnosis of the cases.
	Second, after multiple nucleic acid negative diagnoses, expert response: normal phenomenon, can understand the face of more and more cunning variant strains.
	The virus may not be present at the site of the test.

TextRank (1/6)	Recently, the Changping District of Beijing reported that a woman was diagnosed after 17 nucleic acids were negative in May, which attracted the attention of internet users. Throughout the two years of the epidemic, this kind of event was not an example. After multiple nucleic acids were negative, the diagnosis was still confirmed. Here are the experts' responses.
	As early as August last year, the headquarters for the prevention and control of new corona pneumonia in Ruili City, Yunnan Province, informed a case that had been diagnosed after nucleic acid was negative 13 times before. Then, according to the case flow information, the relevant departments of the Ruili City government adjusted the “health code” of the departing people to the yellow code at night.
	Occasionally, at the beginning of this year, the office of the new coronal pneumonia epidemic prevention and control command of Zhengzhou City also disclosed a similar confirmed case, and the local no. 96 case was finally diagnosed after seven nucleic acid tests for seven consecutive days.
	At the same time, after relevant media investigation, before this, Xi'an has also shown seven nucleic acids after the diagnosis of cases.
	This news makes many people wonder: where is the problem? According to Jiang Qingwu, an epidemiologists and professor at the School of Public Health, Fudan University, it is not the cause of viral variation that has been diagnosed after many nucleic acids, which is more likely to be a problem in the test procedure.
	On 13 May, the patient's nasopharyngeal swab samples (collected on 29 April) were sequenced, and the results showed that the patient was infected with the novel coronavirus Omickrong BA.5 variant.
TextRank + Wor2vec (3/6)	Recently, the Changping District of Beijing reported that a woman was diagnosed after 17 nucleic acids were negative in May, which attracted the attention of internet users. Throughout the two years of the epidemic, this kind of event was not an example. After multiple nucleic acids were negative, the diagnosis was still confirmed. Here are the experts' responses.
	There have been multiple nucleic acid negative confirmed cases through information collection, and it is not difficult to find that multiple nucleic acid negative confirmed cases are not rare.
	Occasionally, at the beginning of this year, the office of the new coronal pneumonia epidemic prevention and control command of Zhengzhou city also disclosed a similar confirmed case, and the local no. 96 case was finally diagnosed after seven nucleic acid tests for seven consecutive days.
	The virus may not be present at the site of the test.
	Jiang Qingwu was interviewed by relevant media. Taking the common throat swab detection method as an example, it is usually only when the virus is discharged from the lung to the throat that it can be detected by the sampling tube.
	He pointed out that the intensity of toxicity and the ability to be detected were two concepts. As long as the virus was objectively present in the detection site, it could be finally detected.

MMR (3/6)	This news makes many people wonder: where is the problem? According to Jiang Qingwu, an epidemiologists and professor at the School of Public Health, Fudan University, it is not the cause of viral variation that has been diagnosed after many nucleic acids, which is more likely to be a problem in the test procedure.
	There have been multiple nucleic acid negative confirmed cases through information collection, and it is not difficult to find that multiple nucleic acid negative confirmed cases are not rare.
	Occasionally, at the beginning of this year, the office of the new coronal pneumonia epidemic prevention and control command of Zhengzhou city also disclosed a similar confirmed case, and the local no. 96 case was finally diagnosed after seven nucleic acid tests for seven consecutive days.
	Third, virus mutation immune escape drive increases or increases the difficulty of nucleic acid screening.
	After 17 times of nucleic acid negative diagnoses, experts responded: The problem may be…
	The virus may not be present at the site of the test.

**Table 2:** Comparison of four automatic summarization methods.

Quantity *P* method	Improved TextRank	TextRank	Word2vec + TextRank	MMR
4	0.400	0.310	0.455	0.435
6	0.590	0.343	0.506	0.483
8	0.657	0.390	0.630	0.527
10	0.610	0.358	0.604	0.546

## Data Availability

The labeled dataset used to support the findings of this study is available from the corresponding author upon request.
